The article "A Comparative Study of Endometriosis and Normal Endometrium Based on Ultrasound Observation" was retracted in 2023. Reasons: signs of a paper mill; suspected computer-generated content; unreliable results or conclusions; concerns about the data.

# A Comparative Study of Endometriosis and Normal Endometrium Based on Ultrasound Observation

**DOI:** 10.1155/2022/7934690

**Published:** 2022-04-30

**Authors:** Lin Jiao, Jue Wang, Lingling Zhu

**Affiliations:** ^1^Department of Ultrasound, Qingdao Chengyang District People's Hospital, Qingdao, 266000 Shandong, China; ^2^Army 73rd Group Military Hospital, Xiamen, 361001 Fujian, China

## Abstract

In order to compare the microscopic ultrastructure of eutopic endometrium and normal endometrium in patients with endometriosis, to study the specific pathogenesis of endometriosis. In this paper, on the basis of using B-ultrasound technology, several patients with endometriosis were subjected to B-ultrasound to observe the ultrastructure of the eutopic uterine endometrium and compared with the pictures of normal endometrium to carry out the specific analysis between the two ultrastructural comparisons. This study is based on the analysis of B-ultrasound images of patients with endometriosis, compares the difference between their ultrastructure and normal human body, and conducts specific pathological diagnosis and analysis to find out the impact of the endometrium in place. The specific factors of the occurrence of lesions and the corresponding treatment methods are proposed. The experimental results show that the ultrastructure of endometriosis eutopic endometrium is different from that of normal endometrium. The microvilli of secretory cells and the cilia of ciliated cells of the former are abnormally increased and lengthened, and they are superior to B-ultrasound technology. The success rate of the examination is 93.75%, which can play an important role in the specific examination process of patients with endometriosis, as one of the actual indicators of detection. Under the electron microscope, microvilli are tiny finger-like protrusions extending from the cell membrane and the cytoplasm on the free surface of the cell, surrounded by the cell membrane and perpendicular to the cell membrane surface.

## 1. Introduction

Severe endometriosis can cause pain and even infertility. Because the pathogenesis is not yet clear, the treatment of endometriosis is difficult. With the continuous development of the current era, various high-tech technical methods are applied in all walks of life. Among them, the high-tech technology applied in the field of medical and health can help doctors carefully observe the lesions that occur in the patient's body, which is a very effective pretreatment diagnostic measure. Medical technology refers to the diagnosis and treatment measures taken by medical institutions and their medical staff for the purpose of diagnosing and treating diseases, making judgments and eliminating diseases, alleviating conditions, alleviating pain, improving functions, prolonging life, and helping patients to restore their health. Endometriosis is a very common gynecological disease, which is different from the endometrial wall of normal women. Most reports claim that women who receive supplemental hormone therapy after menopause also have a higher incidence. In addition, women who give birth relatively late are more frequently affected than women who are born prematurely. Among women of childbearing age, many experts and scholars have made detailed conclusions after a long period of research. A large part of the literature pointed out that with the continuous changes in the environment in recent years, the incidence of this disease has been on the rise compared with 10 years ago. In the 20th century, the understanding of endometriosis has been greatly developed, but there are still many problems that have not been resolved. We even began to question whether Sampson's pathogenesis theory is correct and comprehensive, because it cannot explain why menstrual reflux is common. It is even a physiological phenomenon, and only 10%~15% of women have the disease, which cannot explain multiple, especially distant metastases.

For women, the uterus is a very important reproductive organ. There is a layer of endometrium in the lining of the uterus, which will fall off or thicken under the action of hormones. When the secretion of hormones is abnormal, it may lead to irregular endometrial hyperplasia. Abnormal endometrial hyperplasia, that is, endometriosis, is a common gynecological disease. It is a kind of uterine bleeding disease that will seriously affect the physical and mental health of most women. In recent years, B-ultrasound technology has been used to diagnose abnormal uterine bleeding. The pathogenesis of endometriosis is unclear, but its incidence can be as high as 40%. Women with or without endometriosis have confirmed that there are viable endometrial cells in the female ascites, and the incidence is only about 10%. Endometriosis is caused to a certain extent by the backflow of menstrual blood.

Based on B-ultrasound, by observing the pictures of endometriosis and normal endometrium, the specific manifestations of the disease can be well observed. The corresponding symptoms can be treated to clarify the role of ectopic implantation, that is, the endometrial nature of patients with endometrial dystrophy. This is the key to understanding the pathogenesis of endometriosis, through comparative studies of normal diseases and endometrial hyperplasia.

Endometriosis is the abnormal growth of endometrial tissue and active maturation in the uterine cavity, as well as abnormal growth of other areas covered by mucous membranes. The disease can cause great harm to women and cause serious consequences to women's health. It will affect women's quality of life, and in the long run, there will be great risks. In order to explore the different situations of prokinetic hormone (PROK) 1 and prokinetic receptor (PROKR) 1 in endometriosis, Y Wu and X Wu used quantitative real-time PCR (qPCR) and Western Blot methods. It can detect the expression of PROK 1 and PROKR 1 in endometriosis and normal control endometrial and ectopic endometrium [1]. In order to explore the difference between patients with endometriosis and normal people, Li et al. used pyrosequencing methylation-specific PCR (MSP). It can detect the differences in promoter methylation levels in the three groups of endometrial tissues, which may directly lead to the onset of endometriosis [2]. Endometriosis is considered to be one of the most common causes of female infertility. Medvedev et al. are divided into 3 groups according to the expression of study markers in glands (ER, PGR, Ki-67, BCL-2, and MMP-9) and matrix (ER, PGR, and Ki-67). ER, PGR, and MMP-9 markers established a statistically significant difference between the normal endometrium and the ectopic and ectopic endometrium [3]. Nectin is an immunoglobulin-like adhesion molecule that plays an important role in cell proliferation and tumor metastasis. In order to compare the expression of Nectin-4 in normal endometrial and ectopic endometrial tissues, Bedir et al. speculate that it may be useful to use drugs developed for this molecule to treat endometriosis [4]. Three-dimensional in vitro self-organizing cell cultures called organoids have been developed to study the endometrium and endometriosis. Koninckx et al. simulate the structure of endometrial glandular epithelium and monitor the effects of mitosis, secretion changes, and withdrawal of estrogen and progesterone. They can be used as in vitro models in drug and toxicity testing and disease modeling [5]. In order to study the expression patterns of N-acetylgalactosamine transferase and GalNAc-T6 in clinicopathological features of endometriosis (EMS), Xu et al. obtained ectopic and eutopic endometrial tissue samples from EMS patients and confirmed them with CD-10 immunohistochemistry. The normal control endometrium comes from patients with uterine septum, which may increase the adhesion and invasion of endometrial cells and promote the development of EMS [6]. Endometriosis has been affecting the woman's physical and mental health in recent years. Florova provided data on the abnormal expression of growth factors in patients with endometriosis, the relationship between growth factors and the hormone status in normal and endometrial tissues, and the hypothetical role of growth factors in the pathogenesis of the disease [7]. However, these domestic and foreign research scholars have not carried out theoretically innovative research, have not used professional equipment to observe endometriosis and normal endometrium, and propose specific treatment plans for specific diseases.

Since the beginning of the 21st century, with the continuous iterative update of modern scientific imaging equipment, a wide range of equipment has been used clinically, including electronic computed tomography (CT), computed radiography (CR), direct digital radiography (DR), magnetic resonance, and digital subtraction angiography (DSA). Among them, B-ultrasound is relatively used, which is the main diagnostic measure adopted by most patients in major hospitals. During the actual examination, the B-ultrasound probe was inserted through the vagina and gradually penetrated into the uterus. It can clearly display the patient's uterine cavity, and it can see the patient's uterine contour, uterine cavity endometrium, lesion shape, and other conditions. It is very different from the traditional detection method, which can save the patient's time, so that the doctor can quickly find the cause of the disease and then prescribe the right medicine. The clinical performance of B-ultrasound fully reflects the feasibility of this technique in endometriosis.

## 2. Comparison of Endometriosis and Normal Endometrium

### 2.1. B-Ultrasound Technology

B-Ultrasound intervention technology refers to the puncture of ovarian cysts under the guidance of vaginal ultrasound, and the cyst fluid is extracted, without removing the ovaries, without destroying the normal ovarian tissue, and preserving the reproductive function. It is safe and reliable, does not require hospitalization, has low costs, does not increase the patient's psychological burden, and does not affect the patient's life. Generally, they can go home within two hours after treatment. Ovarian chocolate cyst, ovarian simple cyst, and ovarian crown cyst are suitable for B-ultrasound intervention. B-Ultrasound technology was invented in the 1950s. The sounds that can be heard through the ears in daily life are called sound waves with a frequency of 50 to 10000 Hz. The human ears cannot hear sound waves above 20000 Hz, which are called ultrasonic waves or ultrasonic waves for short. There are two different forms of ultrasound when it is used for diagnosis. One is to diagnose diseases in the form of amplitude. Since the first English letter of amplitude is A, it is called A-ultrasound, also known as one-dimensional ultrasound [8]. The other type of diagnosis in the form of grayscale or brightness is called two-dimensional ultrasound. Because the first English letter of brightness is B, it is also called B-ultrasound, also known as two-dimensional ultrasound or grayscale ultrasound. This method is widely used in the diagnosis of various medical diseases. Ultrasound medicine began in the 1960s, and its development process has undergone four major changes. Ultrasound technology is a high-tech developed in the 20th century. It is a new, multidisciplinary edge science that has attracted widespread attention from scientific and technological workers in the United States, Germany, Canada, Japan, and China. The development of ultrasound technology has opened up new fields for the research of chemical, food, biology, medicine, and other disciplines and has had a significant impact on the abovementioned industries from the application [9, 10]. From traditional A-ultrasound to two-dimensional B-ultrasound, from B-ultrasound to color Doppler ultrasound and continuous technological innovation, ultrasound contrast is one of the most important technologies in the development of ultrasound medicine [11, 12]. In recent years, it has been widely used and clinically recognized. This is the third revolution after two-dimensional Doppler ultrasound and blood flow color imaging, as shown in Figure 1.

Contrast-enhanced ultrasound, also known as contrast-enhanced ultrasound, is a technique that uses contrast agents to enhance backscattered echoes and significantly improve the resolution, sensitivity, and specificity of ultrasound diagnosis. Contrast-enhanced ultrasound is a technology that uses contrast agents to improve echo and significantly improves the resolution, sensitivity, and specificity of diagnostic ultrasound [13]. By improving the performance of related instruments and the emergence of new contrast acoustics, contrast ultrasound can improve two-dimensional ultrasound images and Doppler signals and improve substantial picture imaging of important organs such as the myocardium, liver, kidney, and brain. To a certain extent, it can also reflect the blood flow of these organs, and it can effectively reflect and observe the difference between normal tissues and diseased tissues [14, 15]. Contrast-enhanced ultrasound is a technique that uses contrast agents to enhance the backscatter of the blood, so that the blood flow is clearly displayed, so as to achieve the purpose of differential diagnosis of certain diseases. Since the echo of the contrast agent in the blood is more uniform than the heart wall, and the contrast agent flows with the blood, it is not easy to produce artifacts. Blood flow to tissues has become an important direction for the development of ultrasound diagnosis. In addition to traditional harmonic contrast imaging, contrast ultrasound technology also includes periodic ultrasound imaging, harmonic contrast power imaging, inverse harmonic pulse imaging, low mechanical stimulation imaging, and continuous photographs taken with contrast factors [16]. In any case, the contrast-enhanced ultrasound equipment must have sufficient bandwidth and a high dynamic range. It can provide sufficient parameters, such as MI contrast time and volume. In addition, it must have the ability to save dynamic hard drives in real time. The specific aspects of contrast-enhanced ultrasound are shown in Figure 2.

In the process of doing B-ultrasound, after the image appears, relevant processing must be carried out. There is grayscale processing inside. Grayscale processing refers to the method of changing the gray value of each pixel in the source image point-to-point according to the transformation relationship based on specific target conditions [17, 18]. In grayscale, in the RGB model, if*R* = *G* = *B*, the color represents a grayscale color. The value of *R* = *G* = *B* is called the grayscale value. Therefore, each pixel of the grayscale image only needs one The byte stores the gray value (also called intensity value, brightness value), and the gray range is 0-255. Its purpose is to improve the image quality and make the image appearance clearer. Gray scale scaling is a basic and simple method of spatial image processing in image enhancement processing technology, and it is also an important part of digital software and performance software [19]. Enhancing useful information in an image, which can be a distortion process, is intended to improve the visual effect of an image for a given image's application and purposefully emphasize the global or local characteristics of an image. The grayscale response time is one of the most important concepts, and it plays an important role in the grayscale processing of B-ultrasound, to analyze the factors that affect time and to understand the response time equation, which is as follows:

(1) $$\begin{array}{c} \tau_{r}=\frac{r_{1}d^{2}}{∆\varepsilon \left(V^{2}-V_{th}^{2}\right)}, \end{array}$$

(2) $$\begin{array}{c} \tau_{d}=\frac{r_{1}d^{2}}{∆\varepsilon V_{th}^{2}}. \end{array}$$

Grayscale transformation refers to a method of changing the grayscale value of each pixel in the source image point by point according to a certain target condition and a certain transformation relationship. The purpose is to improve the picture quality and make the display effect of the image clearer. Among them, *A* is the viscosity coefficient of the liquid crystal material, *d* is the cell gap of the liquid crystal cell, and *V* is the starting voltage of the liquid crystal cell.

Gray linear transformation will affect the visual effect of the image to a large extent [20]. The linear transformation can be expressed as

(3) $$\begin{array}{c} \text{g}\left(\text{x},\text{y}\right)=\frac{\text{d}-\text{c}}{\text{b}-\text{a}}\left[\text{f}\left(\text{x},\text{y}\right)-\text{a}\right]+\text{c}. \end{array}$$

When the total number of gray levels of the image is *L*, the distribution of most of the gray levels will not change significantly, while a small part of the excess will have a certain linear change:

(4) $$\begin{array}{c} \text{g}\left(\text{x},\text{y}\right)=\text{c }0\leq \text{f}\left(\text{x},\text{y}\right)<\text{a}, \end{array}$$

(5) $$\begin{array}{c} \text{g}\left(\text{x},\text{y}\right)=\text{d b}<\text{f}\left(\text{x},\text{y}\right)<\text{L},, \end{array}$$

(6) $$\begin{array}{c} \text{g}\left(\text{x},\text{y}\right)=\frac{\text{d}-\text{c}}{\text{b}-\text{a}}\left[\text{f}\left(\text{x},\text{y}\right)-\text{a}\right]+\text{c a}\leq \text{f}\left(\text{x},\text{y}\right)\leq \text{b}. \end{array}$$

When the degree level exceeds a certain interval, the distance can be linearly transformed within a certain interval, and the gray scale beyond this interval can be changed or remain unchanged, as shown in the following formula:

(7) $$\begin{array}{c} \text{g}\left(\text{x},\text{y}\right)=\frac{\text{d}-\text{c}}{\text{b}-\text{a}}\left[\text{f}\left(\text{x},\text{y}\right)-\text{a}\right]+\text{c a}\leq \text{f}\left(\text{x},\text{y}\right)\leq \text{b}, \end{array}$$

(8) $$\begin{array}{c} \text{g}\left(\text{x},\text{y}\right)=\text{f}\left(\text{x},\text{y}\right). \end{array}$$

Gamma correction generally refers to gamma correction. Gamma correction, also known as gamma nonlinearization or gamma coding, is used to perform nonlinear operations or inverse operations on the luminance or tristimulus values of light in a film or imaging system. Gamma correction can be performed after grayscale processing, also known as gamma nonlinearization, which is a nonlinear operation or inverse operation for the grayscale or tristimulus value of light in a film or video system. Gamma correction is defined by the power law formula, as shown below:

(9) $$\begin{array}{c} {\text{V}}_{\text{out}}=\text{A}{\text{V}}_{\text{in}}^{\gamma }. \end{array}$$

The conventional applications in *γ* correction include lightness and gray scale calculation formulas, among which the RGB lightness calculation formula:

(10) $$\begin{array}{c} \text{L}=\sqrt[{2.2}]{\frac{{\left(\text{R}/255\right)}^{2.2}+{\left(1.5\text{G}/255\right)}^{2.2}+{\left(0.6\text{B}/255\right)}^{2.2}}{1+1.5^{2.2}+0.6^{2.2}}.} \end{array}$$

The formula for calculating the brightness after a certain deformation is

(11) $$\begin{array}{c} \text{L}=\text{k}\sqrt[{2.2}]{{\left(\frac{\text{R}}{255}\right)}^{2.2}+{\left(1.5\frac{\text{G}}{255}\right)}^{2.2}+\left(0.6\frac{\text{B}}{255}\right){\left(0.6\frac{\text{B}}{255}\right)}^{2.2}} \end{array}$$

Among them

(12) $$\begin{array}{c} \text{k}=\sqrt[{2.2}]{\frac{1}{1+1.5^{2.2}+0.6^{2.2}}}. \end{array}$$

Linear space generally points to vector space. Vector space, also known as linear space, is one of the central contents and basic concepts of linear algebra. After introducing the concept of vector in analytic geometry, the processing of many problems becomes more concise and clear. The synthesis of the color light brightness follows the physical brightness (linear space), not the brightness that the mind thinks, and the brightness that is synthesized finally needs to be converted to the brightness of the mind, there are

(13) $$\begin{array}{c} {\text{L}}^{2.2}={\text{k}}^{2.2}\left[{\left(\frac{\text{R}}{255}\right)}^{2.2}+{\left(1.5\frac{\text{G}}{255}\right)}^{2.2}+{\left(0.6\frac{\text{B}}{255}\right)}^{2.2}\right], \end{array}$$

(14) $$\begin{array}{c} 1={\text{k}}^{2.2}\left(1+1.5^{2.2}+0.6^{2.2}\right). \end{array}$$

The RGB gray scale calculation formula is

(15) $$\begin{array}{c} \text{Gray}=\sqrt[{2.2}]{\frac{{\text{R}}^{2.2}+{\left(1.5\text{G}\right)}^{2.2}+{\left(0.6\text{B}\right)}^{2.2}}{1+1.5^{2.2}+0.6^{2.2}}}. \end{array}$$

There are many common algorithms for gray scale calculation formulas:

(16) $$\begin{array}{c} \text{Gray}={\text{R}}^{0.299}+{\text{G}}^{0.587}+{\text{B}}^{0.114}, \end{array}$$

(17) $$\begin{array}{c} \text{Gray}=\frac{\left({\text{R}}^{299}+{\text{G}}^{587}+{\text{B}}^{114}+500\right)}{1000}, \end{array}$$

(18) $$\begin{array}{c} \text{Gray}=\left({\text{R}}^{19595}+{\text{G}}^{38469}+{\text{B}}^{7472}\right)\gg 16, \end{array}$$

(19) $$\begin{array}{c} \text{Gray}={\left({\text{R}}^{2.2*0.2973}+{\text{G}}^{2.2*0.6274}+{\text{B}}^{2.2*0.0753}\right)}^{1/2.2}, \end{array}$$

(20) $$\begin{array}{c} \text{Gray}=\frac{\left(\text{r}+\text{g}+\text{b}\right)}{3}. \end{array}$$

Contrast-enhanced ultrasound is the injection of sound contrast agent microbubbles through a peripheral vein. Ultrasound contrast agent is a liquid containing bubbles of a few microns in diameter. Utilizing the characteristics of strong scattering of ultrasonic waves in liquids containing bubbles, clinical ultrasound contrast agents are injected into human blood vessels to enhance the ultrasound Doppler signal of blood flow and improve the clarity and resolution of ultrasound images. The bubbled liquid has strong ultrasonic scattering characteristics, enhances the background of auxiliary resonance, increases the clarity and resolution of the image, and enhances the ultrasonic diagnostic ability [21, 22]. Sensitive and specific ultrasound contrast agents are also called amplifiers. It refers to the addition of microbubbles and other substances in the blood during the ultrasound contrast process at a completely different acoustic impedance value from the blood [23]. The history of using contrast-enhanced ultrasound is quite long. Known ultrasound clarity began in 1968. It mainly relies on salt water with bubbles, because the resolution of microbubbles is better and the retention time is longer, laying the foundation for the development of commercial ultrasound media. The classification of contrast agent products is shown in Figure 3.

### 2.2. Endometriosis

Endometriosis (endometriosis) refers to the development and infiltration of endometrial tissue outside the endometrium. A common gynecological disease in women that occurs when functional endometrial cells is implanted outside the endometrium [24]. If repeated bleeding will cause lumps and nodules, it may cause pain and can invade any part of the body, such as bladder, kidney, ureter, lung, and pleura. But it mainly located in pelvic organs and peritoneum. The most common are the ovaries and uterine ligaments, followed by the uterus and other internal organs, as well as the peritoneum, rectum, and vaginal diaphragm. But because the uterine cavity is connected to the pelvic cavity through the fallopian tube, lesions can affect all pelvic tissues and organs, the most common in ovaries, uterine rectal depression, uterosacral ligament, and other parts, but also can occur in the abdominal cavity, thoracic cavity, limbs, and so on. Therefore, endometrial cells can enter the pelvic cavity through the fallopian tube to grow ectopic. There are many theories about the pathogenesis of the disease. In general, the theory of endometrial implantation is known [25, 26]. This disease mainly occurs in women of childbearing age. The disease does not appear before puberty and ectopic lesions gradually develop and shrinks and degenerates after menopause. The comparison of B-ultrasound pictures of endometriosis (right) and normal endometrium (left) is shown in Figure 4.

The etiology of endometriosis has not yet been elucidated, and the theory of endometrial implantation is generally accepted. In addition, the occurrence of endometriosis may also be related to genetic factors, immune factors, and inflammatory factors. Genetic factors mean that endometriosis has a certain familial clustering. The incidence of some patients may be related to genetics, and the risk of first-degree relatives of patients is 7 times that of no family history. Population studies have found that when one of the twin sisters has endometriosis, the rate of the other can reach 75%. Immune factors refer to abnormal immune regulation. Each link of the occurrence and development of endometriosis plays an important role, which is manifested by the weakened immune surveillance function and the cytotoxic effect of immune killer cells, and the ectopic endometrium cannot be effectively eliminated. Studies have found that endometriosis is related to certain autoimmune diseases, such as systemic lupus erythematosus. Inflammatory factors refer to endometriosis that is also related to subclinical peritonitis. It is manifested by the increase of macrophages, inflammatory cytokines, growth factors, and angiogenesis-promoting substances in the peritoneal fluid. Abnormal content of some factors, or inflammation in the pelvic cavity of the patient, can lead to endometriosis [27].

### 2.3. Comparison of Endometriosis and Normal Endometrium

The uterus of a female individual has an endometrial layer. The endometrial layer refers to a layer of tissue that forms the inner wall of the uterus of mammals. It responds to both estrogen and progesterone. Therefore, it may change significantly with the sexual cycle, which is the estrus cycle, menstrual cycle, and other periods. The endometrium is divided into two layers: the functional layer and the basal layer. Two-thirds of the inner surface of the membrane is the dense layer and the sponge layer. The two are collectively called the functional layer. 2/3 of the inner membrane surface is the dense layer and the sponge layer, collectively referred to as the functional layer, which undergoes periodic changes and falls off under the influence of ovarian sex hormones. The basal layer is the 1/3 of the endometrium close to the myometrium, which is not affected by ovarian sex hormones and does not undergo periodic changes. It undergoes periodic changes under the influence of ovarian sex hormones. The basal layer is the one-third of the endometrium near the myometrium. Its existence is not affected by ovarian sex hormones, nor does it undergo periodic changes. In the initial stage of normal hyperplasia, the supraorbital gland epithelial cells of the endometrial glandular epithelium are the pillars, and uniform morphological cells are neatly arranged on the basement membrane in the glandular cavity. The upper part of the secretory cell is dome-shaped, and the microchip on the free surface is short and straight with a uniform diameter. The upper part of the cytoplasm contains electron density particles of different sizes. The eyelashes located on the empty surface of the eyelashes are short and small. The basic components of a general structure of eyelashes are located in the upper part of the cytoplasm. The space between epithelial cells is narrow, the connections are tight, and the ligaments are visible. Mitochondria in the cytoplasm are oval or elongated. The rough endoplasmic reticulum is scattered, and the reservoir is small and narrow. Free ribosomes are abundant and evenly distributed, and the dispersed Golgi complex nucleus is usually elliptical and located in the center of the cell. There is a smooth outline visible nucleus, showing that the grid cell nucleus is slightly colored and uniform. The details are shown in Figure 5.

Compared with normal endometrium, the ultrastructure of endometrial glandular epithelium in the early stage of endometriosis eutopic hyperplasia is different in the following: The microvilli of secretory cells and cilia of ciliated cells increase abnormally and become longer. Mitochondria in the cytoplasm of epithelial cells increased significantly. The rough endoplasmic reticulum increased and expanded significantly. Lipid droplets and electron-dense particles are common in basement membrane bending.

## 3. Comparative Experiment of Endometriosis and Normal Endometrium Based on B-ultrasound

### 3.1. Based on B-ultrasound Technology Experiment

There are many forms of ultrasound in the diagnosis of diseases: the diagnosis of diseases in the form of amplitude is called “one-dimensional display.” Because the first English letter of the amplitude is A, it is called A-ultrasound, also known as one-dimensional ultrasound. Diagnosing diseases in the form of grayscale or brightness mode is called “two-dimensional display.” Because the first English letter of brightness is B, it is called B-ultrasound, also known as two-dimensional ultrasound or grayscale ultrasound. With the continuous advancement of technology, B-ultrasound technology is now more and more widely used in our medical industry. And with the continuous improvement of the national medical security system, the whole society attaches great importance to the medical industry, the state and individual investment in health is also rising with the continuous growth of the economic level, and related medical imaging equipment has been increasing. And with the continuous iterative update of technology, it is becoming more and more humanized, which meets the needs of most people. After the emergence of a new generation of contrast agents around the world, they have relatively little impact on the human body during the process of being discharged from the body to the outside of the body, and they have very strong safety. Therefore, B-ultrasound technology has been welcomed by the medical industry in many countries at home and abroad. To a certain extent, it has promoted rapid economic and technological growth. The contrast agent market in china has been increasing year by year, and the market size is also increasing year by year. Since 2015, the market size of Chinese contrast agent is shown in Figure 6.

Contrast agents are chemicals injected into human tissues or organs to enhance image viewing. The density of these articles is higher or lower than the surrounding tissue, and the resulting contrast is displayed with certain instruments, such as X-ray observation commonly used iodine preparations and barium sulfate. Contrast agent is a very important part of B-ultrasound operation and provides corresponding basic services for various B-ultrasound instruments. The market demand for contrast agents in China has been very lacking, but compared with the actual strong market demand, most of the contrast agents in China are provided by foreign market shares, accounting for more than 90% of China's total. The supply of domestically produced contrast agents is very limited and cannot keep up with China's market demand. The production level of domestic enterprises is relatively limited, and there is still a lot of room for improvement in the overall R&D level. The specific situation is shown in Table 1.

In 2015, the proportion of foreign capital was 99.50%, and by 2020, the proportion of foreign capital is 96.84%. From the market price point of view, this is because the cost of domestic B-ultrasound contrast agents is very different from that of imported products in terms of product types and scope of use. Most domestic products are used for ultrasound imaging of the heart and blood vessels, while foreign B-ultrasound products are mainly used for B-ultrasound in major hospitals. Included in the related examinations for endometriosis, it is a product positioned close to the civilian population, so the price varies greatly. On average, domestic product prices are relatively high and demand is relatively low. The price of B-ultrasound produced abroad is low, and the demand is relatively small. This is also caused by the inability of domestic product technology. Therefore, marketing promotion is quite difficult. In recent years, as demand has increased, market prices have fallen sharply, as shown in Figure 7

As China's medical industry is becoming more and more developed, the level of related technology continues to increase. The price of China's contrast media products is also declining, and it can gradually keep up with the quality and price of foreign contrast media products. And the demand for contrast agent products in China is increasing. The demand for B-ultrasound contrast agents for the examination of endometriosis alone is increasing year by year, and there is a rising trend. To compare the B-ultrasound pictures of normal endometrium and endometriosis, it is necessary to use a large amount of contrast agent in order to observe the specific pictures well. As shown in Table 2, the number of product segmented demand in China's ultrasound contrast agent market in recent years.

### 3.2. Biological Analysis Experiment of Endometriosis

The basic pathological change of endometriosis is that the ectopic endometrium undergoes periodic bleeding with the changes of ovarian hormones, resulting in the proliferation of surrounding fibrous tissue and the formation of cysts and adhesions, varying purple-brown solid nodules or masses. The clinical manifestations of endometriosis are diverse, the pathological types are complex, and the pathogenesis is unknown. Gynecological examination can be found in the uterine rectal depression, uterosacral ligament, or posterior wall of the cervix, touching one or more hard nodules, such as mung bean or soybean size, and tenderness is obvious. Ectopic lesions of the vagina are mostly located in the posterior fornix, and examination shows that there are tender nodules in the posterior fornix, and in severe cases, it is black and purple. Ovarian hematoma often adheres and fixes to the surrounding area. During examination, a mass with greater tension and tenderness can be palpated, and internal bleeding occurs after rupture, which is manifested as acute abdominal pain. If the degree of pelvic adhesions and the depth of ectopic lesion infiltration are related to hyperthyroidism, the pain of endometriosis is different. In short, we want a standardized assessment of pelvic pain and a comprehensive description of endometrial lesions. It can monitor the related factors that cause pelvic pain and infertility. The degree of adhesion to the pelvic floor can be judged by the following ways to determine the location and severity of the disease. The patient's clinical performance level not only helps to correctly assess the disease state but also provides empirical help for the preoperative assessment of the difficulty of the operation, so that the patient has a more suitable treatment plan, as shown in Table 3.

It is a nonparametric measure of the dependence of two variables. It uses a monotonic equation to evaluate the correlation of two statistical variables. According to the Spearman correlation, the correlation between the degree of pelvic adhesion and the duration can be analyzed. Endometriosis *r* = 0.562, *P* < 0.05, the correlation between pelvic and menstrual adhesion levels *r* = 0.436, *P* < 0.05, depth, lesions, and intraperitoneal. The relationship between different stages of the disease was *r* = 0.726, *P* < 0.05; the relationship between wound depth and menstrual cycle was *r* = 0.637, and *P* < 0.05 was statistically significant. This means that there is a significant positive correlation between the two sets of data. As the clinical distance of endometriosis increases, the level of pelvic adhesions increases, the depth of endometriosis lesions increases, the level of menstruation increases, and the degree of pelvic floor adhesions increases. When the menstrual volume increases, the depth of the endometriosis focus increases, as shown in Figure 8.

The patients with endometriosis and normal people were divided into groups, observing the gap between the B-ultrasound pictures of the endometrium between them, and the test is used to compare the difference in pregnancy between the two groups. Between the control group and the observation group, *Z* = −2,268, *P* = 0.023 < 0.05, indicating that the pregnancy rate of the observation group is obvious, and it can be well observed that the B-ultrasound pictures of patients with endometriosis are very different from those of the normal group. The statistics were significantly higher than the control group (*P* < 0.05), as shown in Figure 9.

In this experiment, 10 patients with ovarian endometriosis were selected, with a total of 20 different parameter standards. The specimens of ectopic endometrial and eutopic endometrial ovarian cysts (2 in the proliferative stage and 8 in the secretory stage) are all from the same place. No drugs and hormone treatment were used before the operation, and the pathology after the operation proved to be endometrial hyperplasia, endometriosis. All samples were taken from samples discarded during elective surgery after sample collection. All experiments have been approved by the ethics committee, and the participating volunteers signed an informed consent form. Another gene is selected from 9 patients with endometrial dystrophy, and the rAFS staging is selected: 2-4 stages, respectively. Eighteen specimens were selected from different patients. They are ectopic endometrium (2 are pelvic wall peritoneum type, 7 are broad ligament type) and ectopic endometrium (5 are proliferative phase, 4 are secretory phase). All samples were taken from samples discarded during elective surgery after sample collection. All experiments have been approved by the ethics committee. Participating volunteers will sign an informed consent form. The specific basic information is shown in Table 4.

### 3.3. B-Ultrasound Contrast Experiment between Endometriosis and Normal Endometrium

Since the sample size in this experiment is less than 50, the normality test of each group of indicators is used. The results showed that the patient's quality of life score conformed to a normal distribution before the relevant examinations. Parametric tests are further quantified, and nonparametric sum tests are used to compare cohorts. The Z indexes are statistical quantities, and the difference is statistically significant with *P* < 0.05. After treatment, it was better than before treatment (*P* < 0.05), the observation group was better than the control group, and the difference was statistically significant (*P* < 0.05). The specific situation is shown in Figure 10.

Endometriosis is a common disease in women. It is uterine bleeding that seriously interferes with the physical and mental health of most women. Patients with endometriosis to the bladder have periodic frequent urination, painful urination, and hematuria. Abdominal wall scars and endometriosis at the umbilical area have periodic local lumps and pain. Patients with intestinal endometriosis may have abdominal pain, diarrhea, or constipation and even have a small amount of blood in the stool periodically. When the ectopic endometrium invades and compresses the ureter, one side of low back pain and hematuria may occur, but it is very rare. In the past few years, B-ultrasound equipment is gradually being used to diagnose the disease, and the diagnostic value is still to be discussed. All patients underwent B-ultrasound and endometrial pathology diagnosis before operation. The doctor observes the pathological diagnosis of the endometrial tissue and compares and analyzes the B-ultrasound of the normal endometrium and the B-ultrasound of patients with endometriosis. The results are shown in Table 5.

## 4. Discussion

Endometriosis is where endometriosis grows outside the lining of the uterus. During menstruation, there is congestion and edema in the long position of endometriosis, causing local pain and easy to cause dysmenorrhea. The main manifestation of endometriosis is abnormal uterine bleeding, such as women with prolonged menstrual periods, menstrual cramps with very frequent menstruation, and bleeding during nonmenstrual periods. This disease often occurs in women of childbearing age who are not pregnant or breastfeeding. If the diagnosis is incorrect, blind treatment can easily delay the patient's optimal treatment time, which delays the treatment of the patient's disease and is likely to cause serious consequences. Therefore, for any reason, abnormal uterine bleeding should be diagnosed before surgery, and finding out the cause of abnormal uterine bleeding provides a reliable basis for establishing a clinical treatment plan. Pathological diagnosis of endometriosis requires better medical equipment and higher medical technology, so it is rarely applied clinically. With the continuous improvement of visual equipment, the clinical application of B-ultrasound equipment has gradually been widely used. Ultrasound is widely used to diagnose uterine diseases. It has the advantages of noninvasiveness and can clearly show the patient's endometriosis, such as the shape of the uterus, endometrium, and pathological changes. There is a significant difference between the B-ultrasound of normal endometrium and the B-ultrasound of patients with endometriosis. B-mode ultrasound is the main inspection method of ultrasound. The development of ultrasound is advancing by leaps and bounds. For example, endoscopic ultrasound, contrast-enhanced ultrasound, three-dimensional imaging, elastography, etc., are all developed on the basis of B-mode ultrasound. Therefore, all physicians and patients undergoing ultrasound work should understand the characteristics of B-mode ultrasound, preparation before examination, examination scope and precautions, etc., in order to better use it to serve the examinee. The success rate of B-ultrasound examination was 93.75%, reflecting the high accuracy of B-ultrasound in the diagnosis of abnormal uterine bleeding. Moreover, it is an observation method performed before the corresponding operation, and it is the first choice for not harming the patient's physical condition.

## 5. Conclusions

At the same time, B-ultrasound is highly praised by the medical community for its convenient operation, fast inspection speed, and clear and dynamic observation of internal organs. In recent years, with the continuous upgrading of medical imaging equipment, various equipment have been widely used in clinical practice. Among them, B-ultrasound is the most widely used equipment, and it shines in the examination of various diseases in medicine. In the specific diagnosis of cervical diseases, B-ultrasound technology is often used for examination. Because B-ultrasound technology has the advantages of noninvasiveness, a B-ultrasound probe can be placed through the vagina, so as to conduct an inspection and analysis of the specific conditions of the patient's uterine cavity and analyze the uterine contour. The endometrium and lesion shape are clearly displayed. Doctors can conduct research and analysis on the specific situation of endometriosis through specific B-ultrasound images and provide guidance for the clinical treatment of patients. In order to explore the difference between the endometrium in patients with endometriosis and the normal endometrium, this study found that there were significant differences between the two in B-ultrasound images after detailed pathological diagnosis. The diagnosis results of endometriosis are consistent with the actual pathological diagnosis results, and the difference between them is not statistically significant, which fully shows that the application of B-ultrasound technology in the diagnosis of endometriosis is very feasible. In the clinical diagnosis of endometriosis, B-ultrasound technology has high diagnostic accuracy and can be used as a specific preoperative diagnosis method for endometriosis.

## Figures and Tables

**Figure 1:** Revolutionary history of contrast-enhanced ultrasound technology.

**Figure 2:** Advantages and applications of contrast-enhanced ultrasound.

**Figure 3:** Contrast agent product classification.

**Figure 4:** Comparison of normal endometrium and endometriosis.

**Figure 5:** The development process of normal uterine wall and ectopic uterine wall.

**Figure 6:** Market size of ultrasound contrast agents in my country in recent years.

**Figure 7:** Product prices of China's ultrasound contrast agent industry in recent years.

**Figure 8:** Correlation between pelvic adhesions and endometriosis.

**Figure 9:** Comparison of pregnancy between the two groups.

**Figure 10:** Two groups of patients undergoing related index test before B-ultrasound test.

**Table 1:** Comparison between foreign-funded contrast agents and domestically produced contrast agents in recent years.

	2015	2016	2017	2018	2019	2020
Foreign-funded contrast agent scale	12139	17590	22800	30192	37789	53650
Domestic contrast agent scale	12200	17800	23200	30892	38700	55400
Percentage of foreign capital	99.50%	98.82%	98.28%	97.73%	97.65%	96.84%

**Table 2:** China's ultrasound contrast agent market segmentation product demand quantity.

	2015	2016	2017	2018	2019	2020
Domestic demand	0.26	0.52	0.93	1.27	2.50	3.64
Foreign investment and imports	33.01	43.25	58.49	76.13	111.73	156.24
Domestic products	0.78%	1.19%	1.57%	1.64%	2.19%	2.30%
Foreign investment and imports	99.22%	98.81%	98.43%	98.36%	97.81%	9.72%

**Table 3:** The relationship between the degree of pelvic adhesion and pain.

Degree of adhesion	Dysmenorrhea				
	*n*	None	Mild	Moderate	Severe
None	40	25	19	4	3
Mild	58	30	31	11	19
Moderate	63	39	37	19	49
Severe	37	24	22	25	35
Hc value	40.91	5.81	2.63	4.27	5.37
*P* value	0.00	0.00	0.02	0.01	0.00

**Table 4:** Basic information table of different experimental subjects.

	GSE7305		GSE11691	
Number of samples	10 pairs		9 pairs	
Different stage	Proliferation phase	Secretory period	Proliferation phase	Secretory period
Number	2	8	5	4
Holding temperature	-80	-80	-80	-80
Keep warm period	3 weeks	3 weeks	3 weeks	3 weeks
Gene chip detection platform	GPL570		GPL96	

**Table 5:** B-Ultrasound diagnosis of endometriosis.

Item	Endometrial pathological diagnosis	B-ultrasound	Diagnosis coincidence rate
Chronic endometritis	33	30	90.91%
Endometrial hyperplasia	28	26	92.86%
Endometrial polyps	26	25	96.15%
Embryo remaining in the uterine cavity	15	15	100%
Uterine fibroids	14	13	92.86%

## Data Availability

No data were used to support this study.
